# The Evaluation Value of CT in the Efficacy of Neoadjuvant Chemotherapy in Ovarian Cancer Patients

**DOI:** 10.1155/2022/7195888

**Published:** 2022-06-08

**Authors:** Daying Mou, Shengyan Xie, Pingyuan Li

**Affiliations:** Department of Gynaecology, The First People,s Hospital of Zunyi, The Third Affiliated Hospital of Zunyi Medical University, Zunyi 563000, Guizhou, China

## Abstract

**Aim:**

To discuss the evaluation value of CT in the efficacy of neoadjuvant chemotherapy in patients with ovarian cancer.

**Methods:**

The clinical, pathological, and CT imaging information of 72 patients with ovarian cancer treated in our hospital from January 2018 to January 2022 were retrospectively analyzed. CT examination and pathological examination were compared to evaluate the efficacy of neoadjuvant chemotherapy.

**Results:**

Using the CRS grading system, 26 cases (36.11%) scored 1, 42 cases (58.33%) scored 2, and 4 cases (5.56%) scored 3. CRS grading system scores of 1, 2, 3, and 4–7 patients were compared, *P* > 0.05. The CT manifestations of lymphadenectasis, degree of peritoneal thickening, ascites, and maximum length diameter of the mass were compared between the patients before and after chemotherapy, *P* < 0.05. According to RECIST 1.1, there were 1 (1.39%) CR, 38 (52.78%) PR, 29 (40.28%) SD, and 4 (5.56%) PD. The comparison was done between RECIST 1.1 and CRS grading system, *P* > 0.05.

**Conclusion:**

CT could be used to evaluate the efficacy of neoadjuvant chemotherapy for ovarian cancer.

## 1. Introduction

As diseases of the female reproductive system, ovarian cancer is a common malignant tumor that occurs in the ovarian region. In China, its incidence rate ranks the third among gynecological malignant tumors, and its death rate tops the list [1, 2]. Epithelial ovarian cancer is the most common type of ovarian cancer, accounting for about 70% of ovarian malignancies [3, 4].

Ovaries being located deep in the pelvic cavity caused early symptoms of epithelial ovarian cancer being difficult to detect. At present, there is still a lack of an effective method for early detection of microscopic pathological changes in ovarian histology. According to the data released by the International Society of Obstetricians and Gynecologists, more than 70% of epithelial ovarian cancers are already at stages III-IV when diagnosed, and the patients have developed abdominal and pelvic metastasis or even distant metastasis [5, 6]. At present, neoadjuvant chemotherapy followed by cytoreductive surgery is the frequently used treatment for epithelial ovarian cancer, but some patients develop chemotherapy resistance and relapse after treatment [7, 8]. So, it is worthy of inquiry for the prognosis of ovarian cancer to judge the efficacy of neoadjuvant chemotherapy as early as possible and select the best time for cytoreductive surgery.

The grading system of the chemotherapy response score (CRS) is the golden criterion for appraising the efficacy of neoadjuvant chemotherapy in ovarian cancer, but its clinical application is limited because of its traumatic nature [9, 10]. Therefore, a noninvasive and effective method to evaluate the efficacy of neoadjuvant chemotherapy is urgently needed. Computerized tomography (CT) is a noninvasive test that looks for tiny changes in any part of the body. The inspection method on the basis of different human body tissue to the different X-ray absorption and transmittance, making use of high sensitivity instrument of human body measurement, the measurement data after the processing of the electronic computer, can produce the inspection area of the section or three-dimensional image, which shows the tiny pathological changes in the inspection area [11, 12]. CT has reached the satisfactory effect in the evaluation of the short-term efficacy of neoadjuvant chemotherapy, but there are few studies on the application of ovarian cancer. Therefore, this study retrospectively analyzed the clinical, pathological, and CT imaging information of 72 patients with ovarian cancer, aiming to analyze the evaluation value of CT in neoadjuvant chemotherapy efficacy for ovarian cancer and provide clinical reference.

## 2. Materials and Methods

### 2.1. Information

The clinical, pathological, and CT imaging information of ovarian cancer patients admitted to our hospital from January 2018 to January 2022 were retrospectively analyzed. Inclusion criteria were as follows: ovarian cancer [13, 14] was pathologically confirmed after cytoreductive surgery, the histological type was epithelial, she was the first diagnosis, and all patients received platinum combined with paclitaxel chemotherapy before cytoreductive surgery. Exclusion criteria were as follows: malignant tumors other than ovarian cancer, incomplete pathological examination results, there were missing items in clinical data and CT imaging data, and CT examination was not performed before and after chemotherapy. Finally, a total of 72 patients were selected, with an average age of (51.26 ± 10.34) years from 34 to 72 years. Clinical data included age, menopausal status, ovarian cancer stage, degree of tumor differentiation, and histological type. CT imaging data included the nature of tumor, lymphadenectasis, invasion of the surrounding tissue, degree of peritoneal thickening, ascites, and maximum length diameter of the mass. This study was approved by the hospital's medical ethics committee and conducted with the informed consent of the patients.

### 2.2. Flow Diagram of the Method

The flow diagram of the method is shown in Figure 1.

### 2.3. Pathological Examination Procedure

After cytoreductive surgery, tissue blocks from the lesion area of epithelial ovarian cancer were taken and fixed in 10% neutral formaldehyde solution, followed by dehydration, paraffin embedding, and sectioning (thickness of 5 *μ*m). Sections were stained with H&E and read by a pathologist.

### 2.4. CT Examination Procedure

All patients were examined by the American GE LightSpeed 64 VCT equipment. Scanning parameters were as follows: tube current 350 mA, tube voltage 120 kV, matrix 512 × 512, layer thickness and layer spacing 5 mm, and 1 mm thin layer reconstruction. Scanning range was as follows: scanned from the diaphragm to the symphysis pubis. Scanning methods were plain scanning and enhanced scanning in arterial and venous phases. In enhanced scanning, the nonionic contrast agent ioversol (300 mgI/mL) was injected intravenously. The injection dose was 1.5 mL/kg, the injection speed was 3 mL/s, and the arterial phase and venous phase scans were performed 30 s and 60 s after injection. Image analysis was conducted independently by two CT diagnostic physicians with titles above deputy director in the blind method. CT findings of patients before and after chemotherapy such as the nature of tumor, lymphadenectasis, invasion of the surrounding tissue, degree of peritoneal thickening, ascites, and maximum length diameter of the mass were observed. Consensus was reached through discussion if differences occurred.

### 2.5. Evaluation of CT Findings

The nature of tumor included solid, solid-cystic, and cystic. Solid means that the solid component accounts for at least 2/3 of the tumor component, solid-cystic means that the cystic component accounts for at least 2/3 of the tumor component, and cystic means that it is between cystic and solid. Lymphadenectasis was determined when the short diameter of the lymph node (measured for 3 times and averaged) was greater than 10 mm. Surrounding tissues include the uterus, bilateral accessories, bladder, ureter, rectum, sigmoid colon, and basin wall. If the CT signs of the patient were indistinct boundaries between masses and tissues, lobulated or irregular thickening of the edges, cloudy, fuzzy or disappeared fatty layer between organs, and uneven mild to moderate enhancement of enhanced scanning, it was judged as invasion of the surrounding tissue; otherwise, it was not invasion of the surrounding tissue. The degree of peritoneal thickening includes grades 1, 2, and 3. Grade 1 was the greater omentum with stained thickening, often with many fine lines and occasionally with a few small nodules, grade 2 was the greater omentum with multiple isolated nodules, and grade 3 was the omentum with nodular thickening fusing with each other, forming “omentum cake sign.” Ascites includes small, medium, and large. The small amount of ascites was defined as a fluid density shadow at the peritoneal reflexes. Medium ascites was defined as uniform crescent-shaped fluid density shadow around the liver, spleen, or bilateral paracolic sulcus. The large amount of ascites was defined as uniform low-density shadows around the abdominal organs, which clustered toward the center under pressure, and the mesangial adipose tissue squeezed it into a circuitous shape. The PACS system was used to measure the maximum length diameter of the mass. The measurement range was the maximum layer of the mass in the axial image. A total of 3 times were measured, and the average value was taken.

## 3. Evaluation Criteria for Neoadjuvant Chemotherapy Efficacy

### 3.1. CT Evaluation Criteria

Evaluation was performed using Response Evaluation Criteria in Solid Tumors 1.1 (RECIST 1.1) [15, 16]. For target lesions, complete remission (CR) referred to the disappearance of all target lesions and the short diameter of pathological lymph nodes was less than 10 mm. Partial remission (PR) referred to the reduction of the sum of the length and diameter of target lesions by at least 30% compared with baseline value. Progressive disease (PD) referred to that the sum of the length and diameter of the target lesions increased by at least 20% over the baseline value and the absolute value increased ≥5 mm or new lesions appeared. Stable disease (SD) referred to that the reduction of the target lesions did not reach PR and the increase did not reach PD.

For nontarget lesions, CR meant that nontarget lesions disappeared and tumor markers returned to the normal level, and the short diameter of lymph nodes was less than 10 mm. Noncomplete remission (non-CR) or nonprogressive disease (non-PD) was the presence of one or more nontarget lesions persisting and/or higher-than-normal levels of tumor markers. PD refers to the presence of one or more new lesions or definite progression of existing nontarget lesions, and an increase in the size of nontarget lesions can lead to increased tumor load. PD referred to the presence of one or more new lesions or definite progression of existing nontarget lesions, and an increase in the size of nontarget lesions could lead to increased tumor load.

After the efficacy evaluation of target and nontarget lesions, the overall efficacy was evaluated. CR: both target and nontarget lesions reached CR, and no new lesions appeared. PR: target lesions reached CR, nontarget lesions reached non-CR or non-PD, and no new lesions appeared; target lesions reached CR, nontarget lesions were not fully evaluated, and no new lesions appeared; target lesions reached PR, nontarget lesions reached non-PD or were not fully evaluated, and no new lesions appeared. SD: target lesions reached SD, nontarget lesions reached non-PD or were not fully evaluated, and no new lesions appeared. PD: if the target or nontarget lesions reached PD, there was no requirement for nontarget lesions and whether there was a new lesion; new lesions appeared, and there was no requirement for target and nontarget lesions; unsuitable for evaluation, incomplete evaluation of target lesions, nontarget lesions to non-PD, and no new lesions.

### 3.2. Pathological Evaluation Criteria

The CRS grading system was used to evaluate the efficacy of neoadjuvant chemotherapy [10, 17]. Score 1: most of the tumors survived, and there was almost no fibrosis-inflammatory reaction or focal fibrosis-inflammatory reaction. Score 2: multifocal or diffuse tumor shrinkage, fibrosis-inflammatory reaction, and survival tumor cells in patchy, small nodular, or multifocal distribution. Score 3: only a small number of residual tumor cells or cell masses, all tumor cells with a total diameter less than 2 mm, or no tumor cells.

### 3.3. Statistical Methods

The data were analyzed by the SPSS 23.0 software, the measurement data conforming to normal distribution were indicated by mean ± standard deviation, and the *t*-test was performed. The counting data were indicated by the number of cases or percentage, carrying out the chi-square test. When the theoretical frequency was less than 5 but greater than 0, the chi-square value should be corrected, and when theoretical frequency was less than 1, the exact probability method was used to calculate. When *P* was less than 0.05, the comparison was considered to be statistically significant.

## 4. Results

### 4.1. Clinical Data Distribution

Among the patients enrolled in this study, the number of patients aged 50–59 was the highest (40.28%), and the proportion of patients aged ≥70 was the lowest (40.28%). Forty cases (55.56%) were postmenopausal and 32 cases (44.44%) were not postmenopausal. Stage IIIC was the highest (58.33%) and stage IIA or IIB was the lowest (4.17%). Six cases (8.33%) were highly differentiated and 66 cases (91.67%) were poorly differentiated. Eleven cases (15.28%) were serous papillary adenocarcinoma, and 61 cases (84.72%) were serous cystadenocarcinoma, as given in Table 1.

The CRS grading system was used to evaluate efficacy. Twenty-six cases (36.11%) scored 1, 42 cases (58.33%) scored 2, and 4 cases (5.56%) scored 3. The comparison result was *P* > 0.05, as given in Table 2.

## 5. CT Findings

The CT manifestations of lymphadenectasis, degree of peritoneal thickening, ascites, and maximum length diameter of the mass were compared between the patients before and after chemotherapy, *P* < 0.05. The above data are given in Table 3 and Figures 2–5.

### 5.1. RECIST 1.1 Evaluation of Efficacy and Its Comparison with the CRS Grading System

According to RECIST 1.1, there were 1 CR (1.39%), 38 PR (52.78%), 29 SD (40.28%), and 4 PD (5.56%). The comparison between RECIST 1.1 and CRS grading system shows that *P* > 0.05 (Table 4). CT images of one patient are shown in Figure 6.

## 6. Discussion

Neoadjuvant chemotherapy plays a crucial part in the treatment of ovarian cancer, and its efficacy directly affects the efficacy of subsequent tumor cell reduction [8, 18]. It is of great significance to accurately appraise the efficacy of neoadjuvant chemotherapy and grasp the optimal therapeutic opportunity of cytoreductive surgery. CT is a noninvasive test that can clearly show small changes in organ tissue. Therefore, this research attempted to appraise the effect of neoadjuvant chemotherapy with epithelial ovarian cancer by CT detection, observe the evaluate effect, and provide guidance for the correct clinical treatment decision of epithelial ovarian cancer.

The results of this research showed that the effect of the RECIST 1.1 evaluation method was indistinguishable from the CRS grading system in the evaluation of neoadjuvant chemotherapy, indicating that the effect of CT examination evaluation was basically the same as that of pathological examination evaluation, which had a certain practicality. It was consistent with relevant research results [19, 20]. In the CT examination results, there were differences in lymphadenectasis, degree of peritoneal thickening, ascites, and maximum length diameter of the mass and were compared between the patients before and after chemotherapy. These results indicated that it was meaningful to evaluate the efficacy of neoadjuvant chemotherapy in CT examination for epithelial ovarian cancer.

The application of this study was to MDCT equipment for scanning the diaphragm to the pubic symphysis, with wide scanning, scanning speed, and scanning layer thickness, in addition to scan image processing software available, more levels in CT image reconstruction, and three-dimensional reconstruction of processing, so as to realize more direction adjustment to make the image clearly show the space of diseased tissue anatomy.

In the process of CT examination, multiphase enhanced scanning can also be carried out to realize the dynamic observation of the relationship between the diseased tissue and blood vessels and adjacent tissues [21]. CT can not only accurately display the location of the tumor but also clearly display the size, shape, density, edge, nature of the tumor, and its impact on the surrounding tissue. It can also provide important information such as tumor blood supply, whether there are swollen lymph nodes, and the degree of enhancement [22]. With the above information, clinicians can more accurately diagnose, stage, treat, and evaluate the efficacy of epithelial ovarian cancer, so that patients can obtain greater treatment benefits.

CT findings of lymphadenectasis in patients with epithelial ovarian cancer showed enlarged, cystic lymph nodes around pelvic iliac vessels, intraperitoneal cavity, and retroperitoneum. Enhanced scan showed uniform or uneven density, marked uniform enhancement, or ring enhancement. After chemotherapy, lymph nodes were significantly reduced, with short diameters generally no more than 10 mm. They were mostly round or oval in shape with smooth sharp edges, clear boundaries, solid, uniform density, and degree of enhancement, and no liquefaction necrosis of the central medulla. These were similar to the results of relevant studies [19, 23].

Ascites usually appears in advanced epithelial ovarian cancer as a result of abdominal pelvic and peritoneal metastasis. The CT findings showed moderate to large amounts of ascites in the abdomen and pelvis. Studies had shown that tumor cells blocking lymphatic vessels is the main mechanism of ascites [24]. For epithelial ovarian cancer patients, ascites provided a microenvironment for tumor cells to survive, which was the material basis for tumor cells' survival, sustained growth, and transplantation [25]. After neoadjuvant chemotherapy, the abdominal fluid volume was reduced and the biological activity of tumor cells was restricted, indicating tumor improvement. Peritoneal thickening was often accompanied by increased ascites, which together with ascites maintain tumor growth. The main CT findings were nodular and irregular patchy thickening around organs or peritoneal surface. CT could clearly display the changes of abdominal water volume and peritoneal thickness before and after neoadjuvant chemotherapy, which was helpful to appraise the efficacy of neoadjuvant chemotherapy [26]. After neoadjuvant chemotherapy, the ovarian cancer mass of the patient subsided, and the maximum length diameter of the mass decreased significantly. The difference of the mass diameter in CT before and after neoadjuvant chemotherapy was significant, and the maximum length diameter of the mass had a reference value for appraising the efficacy of neoadjuvant chemotherapy [12, 22].

However, according to the results of this study, CT had no statistical significance in evaluating the nature of tumor and the invasion of the surrounding tissue before and after neoadjuvant chemotherapy, suggesting that those two CT findings could not provide guidance for evaluating the efficacy of neoadjuvant chemotherapy for epithelial ovarian cancer. Possible reasons are as follows: benign epithelial ovarian cancer masses were usually cystic or cystic-solid, with smooth surface and good mobility, and vesicorectal compression may occur when they become significantly enlarged. Malignant epithelial ovarian cancer tumor was solid or cystic-solid, uneven surface, fixed, and often accompanied by ascites. CT examination was difficult to distinguish the distribution of tumor properties before and after neoadjuvant chemotherapy, so it was not suitable to appraise the efficacy of neoadjuvant chemotherapy by CT examination. In the terminal of epithelial ovarian cancer, tumor often encroaches on surrounding organization and adjacent viscera, the expression was pelvic wall and pelvic bottom peritoneum thickens, the boundary between bump and ovary and uterus was fused mutually, and the adipose gap of lesion periphery was fuzzy. After neoadjuvant chemotherapy, the mass completely subsided, no tumor cells attached to the surrounding tissues and organs of the original tumor, and the signs of tumor invasion were significantly improved. However, it was difficult to avoid tissue fibrosis caused by chemotherapy, which would make CT images show that the fat space between tissues and organs was still a flock-like or cord-like high-density shadow, thus misleading the examiner to judge this CT manifestation as tumor invading surrounding tissues and organs. In addition, the effect of neoadjuvant chemotherapy was not good in some patients, and the mass regression was not obvious. CT examination still showed signs of tumor invasion of surrounding tissues and organs.

By reason of the foregoing, CT findings such as lymphadenectasis, degree of peritoneal thickening, ascites, and maximum length diameter of the mass have significance in appraising the efficacy of neoadjuvant chemotherapy for ovarian cancer, and CT could be used to evaluate the efficacy of neoadjuvant chemotherapy for ovarian cancer.

## Figures and Tables

**Figure 1:** Method' flow diagram. RECIST 1.1, Response Evaluation Criteria in Solid Tumors; CRS, chemotherapy response score grading system.

**Figure 2:** Lymphadenectasis.  ^*∗*^*P* < 0.05.

**Figure 3:** Degree of peritoneal thickening.  ^*∗*^*P* < 0.05.

**Figure 4:** Ascites.  ^*∗*^*P* < 0.05.

**Figure 5:** Maximum length diameter of the mass.  ^*∗*^*P* < 0.05.

**Figure 6:** CT images of one patient. (a)–(c) The CT signs of the patient before treatment. Two small cystic shadows without enhancement are observed in the cervix, about 0.8 cm in diameter. Extensive nodular shadows are observed in the peritoneum, uniform enhancement is observed on enhanced scan, and extensive fluid density shadows are observed in abdominal and pelvic cavities. Extensive fluid accumulation in the abdomen and pelvis. (d)–(f) The CT signs of the patient after treatment. The pelvic mass is significantly reduced, and the pelvic effusion is completely absorbed.

**Table 1:** Clinical data distribution.

Data	Classification	Number of cases	Ratio (%)
Age	<40 years	4	5.56
	40–49 years	19	26.39
	50–59 years	28	38.89
	61–69 years	20	27.78
	≥70 years	1	1.39
Menopausal status	Postmenopausal	40	55.56
	Not postmenopausal	32	44.44
Ovarian cancer stage	Stage IIA or IIB	3	4.17
	Stage IIIA or IIIB	14	19.44
	Stage IIIC	42	58.33
	Stage IVA or IVB	13	18.06
Degree of tumor differentiation	Highly differentiated	6	8.33
	Poorly differentiated	66	91.67
Histological type	Serous papillary adenocarcinoma	11	15.28
	Serous cystadenocarcinoma	61	84.72
	Clear cell adenocarcinoma	0	0

**Table 2:** The CRS grading system used to evaluate efficacy.

Course of treatment	Score 1	Score 2	Score 3	X2	*P*
1 course of treatment	5 (6.94)	4 (5.56)	2 (2.78)	8.440	0.148
2 courses of treatment	10 (13.89)	13 (18.06)	1 (1.39)		
3 courses of treatment	7 (9.72)	20 (27.78)	0 (0)		
4–7 courses of treatment	4 (5.56)	5 (6.94)	1 (1.39)		

**Table 3:** CT findings.

CT findings	Before chemotherapy	After chemotherapy	X2/*t*	*P*
Nature of tumor (*n* (%))			0.608	0.738
Solid	4 (5.56)	4 (5.56)		
Solid-cystic	61 (84.72)	58 (80.56)		
Cystic	7 (9.72)	10 (13.89)		
Lymphadenectasis (*n* (%))			11.403	0.001
Have	33 (45.83)	14 (19.44)		
Not have	39 (54.17)	58 (80.56)		
Invasion of the surrounding tissue (*n* (%))			0.735	0.391
Yes	25 (34.72)	30 (41.67)		
No	47 (65.28)	42(58.33)		
Degree of peritoneal thickening (*n* (%))			22.171	<0.001
Level 1	20 (27.78)	45 (62.50)		
Level 2	43 (59.72)	16 (22.22)		
Level 3	9 (12.50)	11 (15.28)		
Ascites			73.763	<0.001
Not have	0(0)	37 (51.39)		
Small amount	26 (36.11)	25 (34.72)		
Medium amount	24 (33.33)	8 (11.11)		
Large amount	22 (30.56)	2 (2.78)		
Maximum length diameter of the mass (‾*x* ± *s*, cm)	11.26 ± 3.56	8.52 ± 2.28	5.500	<0.001

**Table 4:** RECIST 1.1 evaluation of efficacy and its comparison with the CRS grading system.

CRS grading system	RECIST 1.1				*X* ^2^	*P*
	CR	PR	SD	PD		
Score 1	1	13	8	2	3.832	0.785
Score 2	0	20	18	2		
Score 3	0	5	3	0		

## Data Availability

The data used to support the findings of this study are available from the corresponding author upon request.
